# The Effect of PD-1 Inhibitor Combined with Chemotherapy on the Level of Peripheral Blood T Lymphocytes among Patients with Non-Small-Cell Lung Cancer and Its Relationship with Prognosis

**DOI:** 10.1155/2022/1679191

**Published:** 2022-09-07

**Authors:** Yun Zhao, Jianbo He, Shaozhang Zhou, Ruiling Ning, Wenhua Zhao, Huilin Wang, Cuiyun Su, Wei Jiang, Xiaoning Zhong, Qitao Yu

**Affiliations:** ^1^Department of Respiratory Oncology, Guangxi Medical University Affiliated Tumor Hospital, Nanning, 530021 Guangxi, China; ^2^Pulmonary and Critical Care Medicine, The First Affiliated Hospital of Guangxi Medical University, Nanning, 530021 Guangxi, China

## Abstract

**Objective:**

To explore the effect of combined treatment of PD-1 inhibitor and chemotherapy on the level of peripheral blood T lymphocytes in non-small-cell lung cancer (NSCLC) patients and its relationship with prognosis.

**Methods:**

Retrospective analysis was conducted on 150 NSCLC patients treated in Guangxi Medical University Affiliated Tumor Hospital from June 2018 to September 2020, including 77 patients treated with PD-1 inhibitor combined with chemotherapy as the observation group (OG) and 73 patients with chemotherapy alone as the control group (CG). Therapeutic efficacy, immune function indexes, serum tumor markers, incidence of adverse reactions during hospitalization, 1-year survival rate, and life quality after 6 months of treatment were observed and compared between two groups.

**Results:**

Compared to the CG, the therapeutic effect of OG was evidently better. Six months after treatment, levels of CD4^+^/CD8^+^, NK cells, and CD4 ^+^ in two groups were elevated markedly, and indexes of OG were notably and comparatively higher than those in the other group. After treatment, OG was observed with a marked decline regarding levels of CYFRA21-1, CEA, and CA125 compared to those in the CG; and there was no notable difference in terms of adverse reaction occurrence between two groups, but the 1-year survival rate and 6-month life quality in OG over ranked those in CG.

**Conclusion:**

For NSCLC patients, the PD-1 inhibitor given on the basis of chemotherapy can further improve the clinical efficacy and improve immune function and long-term survival rate of patients on the premise of ensuring the safety of treatment, which is worth promoting in clinical practice.

## 1. Introduction

Lung cancer is one of the most common respiratory system malignant diseases with the number of new cases increasing at a rate of 3% every year, which seriously affects the health of patients [1]. It can be classified into non-small-cell lung cancer (NSCLC) and small-cell lung cancer, and the former takes up more than 80% of all cases with a deadly high mortality rate [2]. The early stage of NSCLC is usually asymptomatic, so 70% to 80% of patients are found to be in an advanced stage at the time of diagnosis [3]. Although early stage patients can be effectively treated with radical surgery combined with drugs, for patients at middle and advanced stage, the best treatment is chemotherapy, which alleviates the disease to a certain extent, improves the life quality, and prolongs life span of patients [4]. Platinum-based chemotherapy has long been the first-line standard treatment for advanced NSCLC patients, but it would inevitably lead to high adverse reaction rate which some patients cannot tolerate, accompanying features of unsatisfactory overall response rate and survival period [5]. Hence, it is urgent and substantial to find a treatment plan with better efficacy and less side effects for NSCLC patients.

In recent years, drugs for tumor-specific immune checkpoint inhibitors have shown great potential. Programmed death-1 (PD-1), one of the cosuppressive molecules of immune cells, can regulate immune system and upgrade self-tolerance by bringing down response of the immune system to human cells and by inhibiting T cell-mediated inflammatory activities [6]. And PD-1 prevents autoimmune diseases and also hinders the immune system from killing cancer cells, making it a novel treatment for advanced NSCLC [7]. However, some studies suggested that the response rate of PD-1 inhibitors alone was only 20% to 40%, from which most patients do not benefit. The changes of natural killer (NK) cells, T lymphocyte subsets, and inhibitory immune checkpoints in patients before and after PD-1 inhibitor treatment require further studies [8].

In the 2021 Chinese Society of Clinical Oncology (CSCO) guidelines, the PD-1 inhibitor combined with chemotherapy is the first-line class IA recommended treatment for patients with NSCLC; however, there are differences in response rates among patients treated with immune checkpoint inhibitors. Therefore, we conducted a related study on the response rate of NSCLC patients treated with inhibitors, as well as the changes in lung function and T lymphocyte subsets in patients before and after treatment. In this study, we included 150 NSCLC patients treated in our hospital from June 2018 to September 2020 and analyzed the efficacy of PD-1 inhibitor combined with chemotherapy in treating NSCLC, hopefully to provide more clinical treatment options for NSCLC patients.

## 2. Materials and Methods

### 2.1. Clinical Information

A retrospective analysis of 150 patients with NSCLC admitted to Guangxi Medical University Affiliated Tumor Hospital from June 2018 to September 2020 includes 82 male and 68 female patients. 77 patients treated with the PD-1 inhibitor combined with chemotherapy served as the observation group (OG), and 73 patients who received chemotherapy alone served as the control group (CG). The following are the inclusion criteria: (1) in line with the NSCLC diagnostic criteria established by the World Health Organization (WHO) via imaging and pathological examinations, (2) patients diagnosed with TNM stage IIIB or IV, and (3) patients with complete case data preservation. The following are the exclusion criteria: (1) patients who have received immunomodulatory therapy, (2) patients with mental illness or disturbance of consciousness, (3) patients with loss of language, cognition, and other functions and inability to communicate, (4) patients with other major physical diseases, (5) patients who have received chemotherapy and radiation therapy before surgery, (6) patients with a survival period of less than 6 months, (7) patients with abnormal liver and kidney function, (8) lactating and pregnant women, and (9) patients with another primary malignancy. This experiment has gained approval from the hospital ethics committee and complies with Helsinki Declaration, with all patients signing written informed consent concerned and their agreement for participation.

### 2.2. Treatment Methods

In the CG group, patients with nonsquamous NSCLC were given carboplatin area under curve 5 and pemetrexed 500 mg/m^2^ in a 3-week cycle for up to six cycles, followed by pemetrexed maintenance, whereas squamous NSCLC were given gemcitabine 1000 mg/m^2^ at days 1 and 8 and cisplatin 75 mg/m^2^ or carboplatin area under curve 5 in a 3-week cycle for up to six cycles, followed by gemcitabine maintenance. On the basis of CG, OG patients were given PD-1 inhibitors by intravenous drip with the treatment of 6 cycles (21 days a cycle). If patients were to experience discomfort and adverse reactions, it should be reported to the superior physician in time with corresponding treatment measures taken.

### 2.3. Observation Indexes

The following are the observation indexes:

1. Therapeutic effect in two groups was assessed and compared according to RECIST evaluation criteria for solid tumors [9]. It is divided into complete response (CR): complete disappearance of lesions was maintained for no less than 4 weeks; partial remission (PR): the sum of tumor lesion radius was reduced by more than 30% and it can be maintained over and above 4 weeks; stable disease (SD): the sum of tumor lesion radii cannot reach PR nor PD; progressive disease (PD): the sum of tumor lesion radii rises by at least 20%, or additional lesions occur; total effective rate = (CR cases + PR cases)/total cases × 100%
2. Immune function indexes were compared between two groups: within 24 hours of admission and after 6 months of treatment, the venous blood was drawn in the morning, and the supernatant was collected at completion of centrifugation and then anticoagulated with EDTA. Later, CD3^+^, CD4^+^, CD8^+^, and CD56 (NK cells) were added to the flow tube to label the cloned monomers, and the serum was added and mixed and then with hemolysin and placed in the dark for 20 minutes. The levels of NK cells, CD4^+^/CD8^+^, and CD3^+^ were detected with a flow cytometer (BD Company, US)
3. Serum tumor markers CYFRA21-1, cytokeratin 19 fragment antigen21-1, carcinoembryonic antigen (CEA), and carbohydrate antigen 125 (CA125) before and after treatment were assessed and compared between two groups. Specifically, a patient's venous blood was taken in the morning, centrifuged at 3000 r/min for 15 min, and levels of CA125, CEA, and CYFRA21-1 were detected by electrochemiluminescence with E170 system produced by Roche Company, Switzerland
4. Occurrence of adverse reactions of two groups during hospitalization was compared, including rash, fever, fatigue, and gastrointestinal symptoms
5. Tumor-free survival rate and 1-year survival rate of two groups were compared. All patients were followed up regularly by returning to the hospital for reexamination, telephone follow-up, text message follow-up, and door-to-door follow-up. The deadline was the death of the patient or March 31, 2022
6. QLQ-C30 quality of life scale [10] was utilized to evaluate a patient's life quality after 6 months of treatment, which includes 5 items of physical, social, emotional, role, and cognitive function. A higher score indicates better quality of life

### 2.4. Statistical Methods

SPSS18.0 (IBM) was used for data analysis, GraphPad Prism 8 (GraphPad Software) for figures attached, log-rank analysis for survival analysis, and Kaplan-Meier for survival curve. A chi-square test was applied for the analysis of enumeration data, and Student's *t*-test was for comparison of measurement data. And *P* < 0.05 was taken to be statistically different.

## 3. Results

### 3.1. General Information Comparison

No marked differences were observed regarding gender, age, and smoking history between two groups, and subjects were comparable (*P* > 0.05, Table 1).

### 3.2. Comparison of Therapeutic Efficacy

The numbers of patients assessed with CR, PR, SD, and DP in OG were 0, 41, 29, and 7, respectively. And corresponding data in CG were 0, 26, 20, and 27, respectively. Statistically, OG held a strikingly higher total effective rate of treatment than that in CG (*P* < 0.05, 53.25% *vs.* 35.62%, Table 2).

### 3.3. Comparison of Immune Function Indexes

Before treatment, no marked difference was observed in levels of CD4^+^/CD8^+^, CD8^+^, CD4^+^, and NK cells between two groups (*P* > 0.05), while six months after treatment, despite CD8^+^ having few fluctuations, levels of CD4^+^/CD8^+^, CD8^+^, CD4^+^, and NK cells were upregulated evidently (*P* < 0.05), and the increase in OG was markedly higher than those in OG (*P* < 0.05, Figure 1).

### 3.4. Comparison of Serum Tumor Markers before and after Treatment between Two Groups

Before treatment, no evident difference was observed regarding serum tumor marker levels between two groups (*P* > 0.05), while levels of CYFRA21-1, CEA, and CA125 of both groups were downregulated after treatment. In addition, indicators in OG were markedly lower than those in CG (*P* < 0.05, Figure 2).

### 3.5. Comparison of the Incidence of Adverse Reactions

The number of patients in OG who developed rash, fever, fatigue, and gastrointestinal symptoms was 3, 3, 4, and 5, respectively. Those in CG were 4, 4, 3, and 3, respectively, showing no marked difference in terms of incidence of adverse reactions when compared with that of OG (*P* > 0.05, 19.48% vs. 19.18%, Table 3). The adverse reactions of patients were treated symptomatically during the treatment and were effectively alleviated afterwards.

### 3.6. Comparison of 1-Year Survival Rate

The overall survival curve analysis indicated that OG patients possessed a markedly higher 1-year overall survival rate than OG (68.83% (53/77) vs. 49.32% (36/73)) (*P* < 0.05, Figure 3).

### 3.7. Comparison of Life Quality 6 Months Posttreatment

Compared with CG, the scores of physical, role, emotion, cognition, and social dimensions of life quality in OG were markedly improved after treatment (*P* < 0.05, Table 4).

## 4. Discussion

With changes in social environment and life pressure, the incidence of lung cancer is getting higher and younger [11]. In recent years, chemotherapy has gradually become an important method for the treatment of NSCLC and has achieved good therapeutic effects. However, some patients have to forgo treatment due to multiple adverse reactions of chemotherapy [12]. Therefore, finding new treatment options is of great clinical significance. With the continuous development of molecular biology techniques, a growing number of molecular biological targets are being used in the treatment of NSCLC and have been proved to have positive therapeutic effects. PD-1, an important immunosuppressive molecule and a member of the immunoglobulin superfamily, which is one of those targets [13]. Studies have found that immunomodulation targeting PD-1 was of great significance in fighting infections, autoimmune diseases, and tumors, as well as promoting the survival of transplanted organs [14]. Although the efficacy of PD-1 has been affirmed in the past, few studies have focused on the comprehensive impact of PD-1 combined with chemotherapy on NSCLC patients.

In this study, we first observed that OG patients possessed much higher total effective rate than that in CG, indicating that combined treatment of PD-1 inhibitor and chemotherapy performed better regarding short-term efficacy in the treatment of NSCLC patients. Clinically, changes of NK cells and T lymphocyte subsets are used as indicators of immune status and prognosis in NSCLC patients. CD4^+^ is mainly a helper T lymphocyte that can promote the antitumor effect of effector cells, and CD8^+^ is an inhibitory T lymphocyte. The two generally maintain a balanced state [15]. A study [16] has shown that the proportion of immune subsets of peripheral blood lymphocytes in lung cancer patients was abnormal, which suggested that the immune function of patients was unbalanced. However, the increase of CD8^+^ cells was the basis of cellular immune damage, and the decline of CD4^+^ cells could cause immune escape of tumor cells [17]. Results of present study suggested that CD4^+^, CD4^+^/CD8^+^, and NK cells in both groups went markedly higher after treatment, and it was notable that OG held much vivid improvement on these indicators when compared to CG, indicating that the PD-1 inhibitor combined with chemotherapy could more effectively improve the immune function of NSCLC patients than chemotherapy alone. A former study [18] found that the proportion of immune subsets of peripheral blood lymphocytes may be abnormal in NSCLC patients, of whom the peripheral blood CD8^+^ cells increased, CD4^+^ cells decreased, CD4^+^/CD8^+^ decreased, and tumor cells occurred immune escape. When the tumor burden was relieved, the abnormal lymphocyte subsets could gradually recover, which is similar to our observations. The reason for the enhanced immune function of patients in our study may also be that the PD-1 inhibitor relieving the inhibitory effect of immune checkpoints activated T lymphocytes with killing effect, thereby enhancing the immune ability and antitumor ability of the body. In addition, a study [19] showed that in the course of NSCLC, the apoptosis of tumor-specific T cells was mediated by PD-1-dependent and independent mechanisms, and the PD-1-dependent mechanism could promote the immune escape of tumor cells in NSCLC patients. This could also explain our observations.

Serum tumor markers CYFRA21-1, CEA, and CA125 are closely related to the disease progression and prognosis of NSCLC, and elevated levels of tumor markers indicate poor prognosis and short survival time. CYFRA21-1 is the most valuable serum tumor marker for NSCLC detection, a soluble acidic protein of cytokeratin detected by monoclonal antibody, and is mainly distributed in the cancerous breast and lung epithelium and released into the blood, which is of essential clinical value in judging the efficacy of NSCLC [20, 21]. CEA is a class of acidic glycoproteins located in hollow organs such as the respiratory tract and digestive tract and consists of sugar chains and peptide chains. It exists in macrophages, monocytes, and multinucleated cells, has human embryonic epitopes, and is specific for tumor-associated antigens that are associated with tumor recurrence [22]. CA125 is a class of tumor carbohydrate antigens with high concentrations in malignant tissues and tumor cells and can be released into the blood when tumor tissues are destroyed, which is of great value in the diagnosis and prognosis of NSCLC [23]. Results of our study showed that CYFRA21-1, CEA, and CA125 in both groups all declined after treatment, and the decrease in OG was even marked, suggesting that the PD-1 inhibitor combined with chemotherapy in NSCLC treatment could better and effectively alleviate the disease than that of chemotherapy alone. In addition, long-term prognosis results of two groups showed that the 1-year overall survival rate in OG was notably higher than that in CG. This is also in line with our previous conclusion that “PD-1 inhibitor combined with chemotherapy in the treatment of NSCLC could be more effective than chemotherapy alone.” This result also showed that PD-1 did not markedly increase the related adverse reactions in patients receiving chemotherapy, suggesting that PD-1 inhibitors were generally well tolerated in NSCLC patients. Finally, we compared the life quality between two groups after treatment, and the results showed that OG patients rated a more satisfactory quality of life.

## 5. Conclusion

To sum up, for NSCLC patients, the PD-1 inhibitor on the basis of chemotherapy could further improve the clinical efficacy, as well as the immune function and long-term survival rate of patients on the premise of ensuring the safety of treatment, which is worthy of promotion in clinical practice. However, this study still has certain shortcomings, such as a dearth of detection of PD-L1 expression status and relevant information on the basic lung status of the patient, which may have a certain impact on the results of lung function. Due to the small sample size and limited observation time, more rigorous large-sample clinical trials are still needed in follow-up studies.

## Figures and Tables

**Figure 1:** Comparison of immune function indicators between two groups; (a) comparison of CD4^+^ between two groups before and after treatment; (b) comparison of CD8^+^ between two groups before and after treatment; (c) comparison of CD4^+^/CD8^+^ between two groups before and after treatment; (d) comparison of NK cells between two groups before and after treatment. When comparing between groups or before and after treatment within a group, ∗ indicates *P* < 0.05.

**Figure 2:** Comparison of serum tumor markers in two groups before and after treatment; (a) comparison of CYFRA21-1 between two groups before and after treatment; (b) comparison of CEA between two groups before and after treatment; (c) comparison of CA125 between two groups before and after treatment. ∗ indicates *P* < 0.05.

**Figure 3:** Comparison of 1-year survival rate; ∗ indicates *P* < 0.05.

**Table 1:** Comparison of general information [*n* (%)].

Factors	Observation group (*n* = 77)	Control group (*n* = 73)	*t*/*χ*^2^	*P*
Gender			0.024	0.877
Male	40 (51.95)	37 (50.68)		
Female	37 (48.05)	36 (49.32)		
Age (years)			0.110	0.701
≤61	38 (49.35)	38 (52.05)		
>61	39 (50.65)	35 (47.95)		
BMI (kg/m^2^)			0.036	0.849
≤23	41 (53.25)	40 (54.79)		
>23	36 (46.75)	33 (45.21)		
History of smoking			0.019	0.891
Yes	42 (54.55)	39 (53.42)		
No	35 (45.45)	34 (46.58)		
Clinical stage			0.001	0.983
Stage IIIB	36 (46.75)	34 (46.58)		
Stage IV	41 (53.25)	39 (53.42)		
Pathological type			0.057	0.972
Squamous cell carcinoma	21 (27.27)	19 (26.03)		
Adenocarcinoma	46 (59.74)	45 (61.64)		
Others	10 (12.99)	9 (12.33)		
Tumor location			0.036	0.849
Left lung	41 (53.25)	40 (54.79)		
Right lung	36 (46.75)	33 (45.21)		

**Table 2:** Comparison of therapeutic efficacy [*n* (%)].

Therapeutic effect	Observation group (*n* = 77)	Control group (*n* = 73)	*χ* ^2^	*P*
Complete remission	0	0	—	—
Partial remission	41 (53.25)	26 (35.62)	—	—
Stable disease	29 (37.66)	20 (27.40)	—	—
Disease progression	7 (9.09)	27 (36.99)	—	—
Total effective rate	41 (53.25)	26 (35.62)	9.499	0.002

**Table 3:** Comparison of incidence of adverse reactions [*n* (%)].

Complications	Observation group (*n* = 77)	Control group (*n* = 73)	*χ* ^2^	*P*
Rash	3 (3.90)	4 (5.48)	—	—
Fever	3 (3.90)	4 (5.48)	—	—
Fatigue	4 (5.19)	3 (4.11)	—	—
Gastrointestinal symptoms	5 (6.49)	3 (4.11)	—	—
Incidence of adverse reactions	15 (19.48)	14 (19.18)	0.002	0.963

**Table 4:** Comparison of quality of life.

Factors	Observation group (*n* = 77)	Control group (*n* = 73)	*t*	*P*
Physical function	72.74 ± 2.75	61.91 ± 1.15	31.16	<0.001
Role function	71.12 ± 2.39	62.44 ± 1.44	26.76	<0.001
Emotional function	72.42 ± 2.3	62.09 ± 1.36	33.25	<0.001
Cognition function	72.03 ± 2.26	62.18 ± 1.24	32.84	<0.001
Social function	72.04 ± 2.21	62.4 ± 1.43	31.53	<0.001

## Data Availability

The labeled dataset used to support the findings of this study is available from the corresponding authors upon request.
